The article "Application of Amiodarone and Cedilan in the Treatment of Patients with Arrhythmia after Esophageal and Lung Cancer" was retracted in 2023. Reasons: signs of a paper mill; compromised peer review; unreliable results or conclusions.

# Application of Amiodarone and Cedilan in the Treatment of Patients with Arrhythmia after Esophageal and Lung Cancer

**DOI:** 10.1155/2023/8026918

**Published:** 2023-04-13

**Authors:** Hongjin Ge

**Affiliations:** Department of Thoracic Surgery, Tianchang People's Hospital, Tianchang, Anhui Province, China

## Abstract

**Objective:**

To explore the effect of amiodarone and cedilan in the treatment of patients with arrhythmia after esophageal and lung cancer.

**Methods:**

The data of 60 patients with postoperative complications of arrhythmias after esophageal and lung cancer from January 2018 to July 2021 were retrospectively analyzed and divided into an observation group (*n* = 30) and control group (*n* = 30) according to the random number grouping principle. The former group was treated with amiodarone, and the latter group received cedilan.

**Results:**

The effective rate of treatment was significantly higher in the observation group than the control group (*P* < 0.05). The observation group had the drug onset time obviously shorter than the control group (*P* < 0.001). The average ventricular rate after treatment in the observation group was remarkably lower than the control group (*P* < 0.001). The observation group exhibited obviously better cardiac function after treatment as compared to the control group (*P* < 0.05). The incidence of adverse reactions in the observation group was notably lower than the control group (*P* < 0.05). Moreover, the observation group had less stress after treatment than the control group (*P* < 0.001). The blood pressure level of the observation group after treatment was significantly better than the control group (*P* < 0.05).

**Conclusion:**

Amiodarone can relieve stress in patients with arrhythmia following esophageal and lung cancer surgery, stabilize blood pressure, and mitigate arrhythmia symptoms. Our findings are worthy of promotion and application in clinic.

## 1. Introduction

Lung cancer, as a highly prevalent malignant tumor whose etiology has not been completely clarified, presents with complex clinical manifestations. In the early stage, patients do not experience any discomfort or the symptoms and signs lack specificity, and most patients are diagnosed with advanced disease, with a high clinical prevalence and death rate. Esophageal cancer is a malignant tumor of the digestive tract, which may occur in all segments of the esophageal mucosa, with a higher incidence in male than in female [1]. At this stage, surgery is an effective treatment for esophageal cancer, but radical surgery for esophageal cancer is complicated and time-consuming, which will cause greater trauma to patients and yield a higher chance of postoperative complications. Esophageal and lung cancer generally require surgical treatment, and anesthesia, hypoxic acidosis, sudden blood pressure fluctuations, traction trauma, and stress response during thoracotomy are all major causes of postoperative complications [1, 2]. Early patients are prone to arrhythmias that persist for a long time and remain complicated to remedy [3], and later, they may suffer from decreased circulatory function and cardiac arrest [4, 5], which can seriously affect the postoperative recovery process. According to the World Health Organization (WHO), the probability of postoperative arrhythmia is approximately 0.8% to 54.2% after lung cancer [6], while the probability of postoperative arrhythmia is 2.6% to 29.8% after esophageal cancer [7]. Furthermore, in certain preoperative patients with circulatory system illnesses, cardiopulmonary performance diminishes dramatically, and the incidence of arrhythmia increases significantly. As a result, failure to intervene on time may result in death [8].

At present, the drugs used to treat arrhythmia are mainly sodium channel blockers, *β*-adrenergic receptor blockers, calcium channel blockers, and repolarization process extension drugs [9]. Cedilan is a popular digitalis medicine that helps relieve arrhythmia symptoms in patients; however, it might produce gastrointestinal problems, and patients are at risk of digitalis poisoning [10]. Some studies have found that amiodarone can reduce the average ventricular rate of patients with arrhythmia more quickly than cedilan and relieve their stress state [11, 12]. Taken together, the reason behind a fairly favorable therapeutic effect of amiodarone is that it has no inhibitory effect on the patient's left ventricular function and is beneficial in protecting the patient's cardiac function.

A review of previous literature reveals no studies on the use of amiodarone and sildiran in patients with postoperative arrhythmias in esophageal and lung cancer. In recent years, with the widespread application of Chinese medicine in the treatment of this disease, it has been found that Chinese medicine has obvious advantages in long-term medication and control of clinical symptoms, featuring individualized treatment, diverse formulae, and significant efficacy, and the combination with western medicine can greatly improve the therapeutic effect. Chinese medicine adopts a holistic concept and treats the disease with evidence. It is believed that the overall pathological changes of the disease are based on the deficiency of the heart and the deficiency of the qi, and the cause of the disease is related to the deficiency of the heart and qi. Nourishing the heart, benefiting qi, and opening up the blood vessels are the main treatment principles. As a result, we aimed to investigate the effect of combining the two on patients with arrhythmia following esophageal cancer and lung cancer surgery. We evaluated the drug by observing routine indicators of arrhythmia.

Furthermore, we investigated the efficacy of amiodarone and cedilan in the therapy of arrhythmias in patients with esophageal and lung cancer. According to the findings of this study, the most common adverse effects of the two groups of patients were dizziness, weariness, and gastrointestinal symptoms. The observation group had obviously lower adverse reaction rate than the control group, suggesting that such a combination can be used in middle-aged and elderly patients with lung and esophageal cancer. Following are the main contributions:

- To explore the effect of amiodarone and cedilan in the treatment of patients
- To explore the effect of combination of the two on patients with arrhythmia after operation of esophageal and lung cancer
- To compare the treatment effect, average ventricular rate, onset time, cardiac function, and incidence of adverse reactions, stress indicators, blood pressure levels between the two groups

The rest of the paper was organized as follows: in section 2, we offer an overview of the materials and methods.  Section 3 is about the datasets and evaluation metrics. Moreover, the experimental details were also presented. In Section 4, results are discussed. Finally, the conclusion is presented in Section 5.

## 2. Materials and Methods

### 2.1. Research Design

This study, a controlled study, was conducted in our hospital from January 2018 to July 2021, which was intended to explore the application effects of amiodarone and cedilan in the treatment of patients with postoperative arrhythmia after esophageal cancer and lung cancer.

The randomization was carried out using an online web-based randomization tool (https://www.randomizer.org/). The original sample size calculation estimated that 30 patients in each group would be needed to detect a 3-point difference between groups in a 2-sided significance test with a power of 0.8 and an alpha error level of 0.05.

Informed consent was obtained from patients and signed prior to enrollment in this study. The study protocol was approved by the hospital ethics committee. Ethics number: SD-SD20180102. All processes were in accordance with the Declaration of Helsinki.

### 2.2. Recruitment of Research Objects

The data of patients with postoperative complications of arrhythmias after esophageal and lung cancer in our hospital from January 2018 to July 2021 were retrospectively analyzed, and patients were included according to the following criteria. (1) The patient was diagnosed as esophagus cancer/lung cancer by imaging and pathological examinations [13, 14] and given surgical treatment, and arrhythmia of more than 3 minutes consistently occurs within 7 days after operation (the arrhythmia is diagnosed based on the 6^th^ edition *Diagnostics* [15] of People's Medical Publishing House); (2) the patient was treated in this hospital for the whole course, and there was no death, transfer to the hospital or stopping treatment; (3) the clinical data of the patient was completed. Similarly, patients were excluded according to the following criteria: (1) patients who were unable to communicate with them due to hearing, language impairment, mental illness, or unconsciousness; (2) patients who withdrew from treatment, died, had treatment plans changed, or lost to follow-up; (3) the same type of arrhythmia existed before treatment, which is not clear that it is caused by surgery or postoperative factors; and (4) patients complicated with other serious organic diseases.

### 2.3. Procedures

A total of 60 patients were included in the present study, and they were randomly divided into the observation (*n* = 30) and the control (*n* = 30). On the same day, the patients agreed to participate in the study, and the study team collected social demographic statistics. According to the analyses, no statistically significant difference was noted in the general data of the two groups (*P* > 0.05), see details in Table 1.

### 2.4. Moral Considerations

This study was compiled in accordance with the principles of the Declaration of Helsinki [16] and was approved by the ethical committee of the hospital. The patients were recruited, to whom the research team explained the objective, significance, content, and confidentiality of the study they enrolled in, and the informed consent form was obtained subsequently.

### 2.5. Withdrawal Criteria

In cases where the research team judged it inappropriate to continue the experiment, their case records were retained but data analysis was not performed if the following conditions occurred: (i) adverse events or severe adverse events; (ii) illnesses deterioration during the experiment.; (iii) severe complications; (iv) unwilling to continue the clinical trial and requests to withdraw from the clinical trial.

### 2.6. Methods

The observation group was treated with the amiodarone (Shan Dongfangming Pharmaceutical Group Co., Ltd., Zhunzi H20044923). 150 mg amiodarone was added to 10 mL of 5% glucose solution for intravenous injection. If the initial loading dose is not obvious, an additional dose of 150 mg was added within 15 minutes, followed by continuous intravenous infusion at 0.5–1 mg/min, with a total dose of ≤1.2 g in 24 hours.

The control group was treated with the cedilan. If the patient had not used digitalis in the past 7 days, then 0.4 mg cedilan (Shanghai Zhaohui Pharmaceutical Co., Ltd., SFDA approval no. H31021178) was added to 20 mL of 5% glucose solution for intravenous injection, 0.4 mg was added for those who were ineffective within 30 minutes, and 0.2 mg for those who were still ineffective, and the total dose was 1 mg. If the patient had used digitalis within the past 7 days, 0.2 mg cedilan was given as an intravenous bolus, 0.2 mg was added for those who were ineffective within 30 minutes, and 0.2 mg was added for those who were still ineffective, and the total dose was 0.6 mg.

Electrocardiograms and blood pressure were monitored continuously in both groups before and after dosing. If patients converted to sinus rhythm or had a heart rate decrease to 70 beats per minute during intravenous administration, the drug was discontinued. In addition, blood pressure was immediately measured, and a 12-lead ECG was recorded.

The two groups were treated with Yangxin Yiqi Tongmai decoction: 15 g Radix Astragali, 12 g *Codonopsis pilosula*, 9 g *Panax quinquefolius*, 9 g Radix Pseudostellariae, 15 g Radix Rehmanniae, 12 g Radix Ophiopogonis, 9 g *Schisandra chinensis*, 12 g Radix Glycyrrhizae, 15 g *Salvia miltiorrhiza*, 15 g Szechuan Lovage Rhizome, 15 g *Achyranthes bidentata*, 15 g Radix *Achyranthes bidentata*, 9 g Ramulus Cinnamomi, 5 g Aconite, 9 g dried ginger, 12 g Semen Ziziphi Spinosae, and 15 g Platycladi Seed. The above medicine was decocted in water, one dose daily, taken in morning and evening, for a total of 1 month.

### 2.7. Observation Criteria

1. *General data*: the general information sheet is self-made and includes the frequency of hospitalization, name, gender, age, weight, BMI, marital status, education level, place of residence, income level, medical payment method, lifestyle habits, and type of disease.
2. *Clinical symptoms*: patients were considered significantly effective if their clinical symptoms largely disappeared and converted to sinus rhythm, or if the ventricular rate decreased to 100 beats/min within 15 minutes of dosing. Similarly, patients were considered effective if their symptoms improved and converted to sinus rhythm within 15–30 minutes of dosing, or if their ventricular rate decreased ≥20% from baseline values. In addition, patients were considered ineffective if their symptoms did not improve after 30 minutes of dosing and did not meet the criteria for apparent effectiveness.
3. *Average ventricular rate and onset time*: the average ventricular rate and onset time of the drugs in the two groups were recorded.
4. *Cardiac function*: at pre- and post-treatment, patients were placed in the supine position, and apical four-chamber color Doppler ultrasonography (GE Medical Voluson P6, National Instruments No. 20152062178) was performed to examine left ventricular end-diastolic diameter (LVEDD), left ventricular ejection fraction (LVEF), and cardiac output per beat (SV).
5. *The incidence of adverse reactions*: adverse reactions ranged from dizziness, fatigue, gastrointestinal reactions, elevated creatinine, and elevated blood phosphorus. The number of patients with adverse reactions was counted.
6. *Stress indicators*: after treatment, 5 ml of fasting peripheral venous blood was collected from the patient in the morning and centrifuged at 3000 r/min for 15 min, and then the serum was isolated. The enzyme-linked immunosorbent assay (Beijing Kewei Clinical Diagnostic Reagent Co., Ltd., Enzyme Combined immunosorbent kit, S20060028) was used to measure blood sugar level and insulin level.
7. *Blood pressure level*: patients were required to sit in meditation for 10 minutes before and after the treatment to ensure that they did not smoke or consume caffeine before the blood pressure test. Measurements were performed using a standard mercury column sphygmomanometer (Jiangsu Yuyue Medical Equipment Co., Ltd., Su Yi No.: 20152070945). Measurements were taken with the patient in a sitting position, with both legs naturally flat. The lower edge of the cuff was approximately 2 cm from the anterior midline of the elbow. The balloon tube was facing the brachial pulse. The blood pressure in the patient's upper arm was recorded, and the mean value was recorded.

### 2.8. Statistical Analysis

The data analysis was conducted using SPSS 20.0, and GraphPad Prism 7 (GraphPad Software, San Diego, USA) was utilized for graphics plotting. The results included counting data and measurement data, which were analyzed by X^2^ and the *t*-test, respectively. *P* < 0.05 indicates statistically significant difference.

## 3. Results

### 3.1. Intergroup Comparison of the General Data

In terms of general data, no statistical difference was observed between the two groups (*P* > 0.05). See Table 1.

### 3.2. InterGroup Comparison of Treatment Effects

The observation group had a much higher effective rate of treatment than the control group (*P* < 0.05). See Figure 1.

### 3.3. InterGroup Comparison of Average Ventricular Rate and Onset Time

After treatment, the observation group exhibited medication onset time and average ventricular rate obviously lower than the control group (*P* < 0.001). See Figures 2 and 3.

### 3.4. InterGroup Comparison of Heart Function

The observation group exhibited obviously improved cardiac function after treatment when compared to the control group (*P* < 0.05). See Table 2.

### 3.5. InterGroup Comparison of the Incidence of Adverse Reactions

The incidence of adverse responses was considerably lower in the observation group than the control group, with statistically significant difference (*P* < 0.05, Table 3).

### 3.6. InterGroup Comparison of Stress Indicators

The stress indicators were noticeably better in the observation group after the treatment than the control group (*P* < 0.001) for the whole process, as shown in Figure 4.

### 3.7. InterGroup Comparison of Blood Pressure Levels

Following treatment, the observation group had blood pressure level significantly lower than the control group (*P* < 0.05). See Table 4.

## 4. Discussion

Arrhythmias are defined as changes in the formation of cardiac impulses and abnormalities in the conduction of heart rate and rhythm. The main mechanisms underlying them are abnormal autonomic, reentrant, and triggered activity [17, 18], and patients with severe arrhythmias usually experience rapid onset, and their hemodynamic indices are already markedly altered, in which they face a serious risk of death. In etiological terms, arrhythmias is mainly classified into hereditary arrhythmias and acquired arrhythmias. Hereditary arrhythmias is mostly caused by mutations in gene channels, while acquired arrhythmias can originate from various organic heart diseases [19, 20]. The incidence of arrhythmias would be elevated in patients subjected to anesthesia, hypothermia, and thoracotomy.

The esophagus is the narrowest part of the digestive tract, and its physiological anatomical location is closely intertwined with the respiratory tract. Esophageal cancer is a highly prevalent clinical malignant tumor of the digestive tract. Surgery is an effective method to treat esophageal cancer at this stage, but the postoperative complications are prone to endanger patients' life. Lung cancer is also prone to some postoperative complications, such as respiratory failure, as well [21, 22]. Surgery is currently the primary modality for treating patients with esophageal and lung cancers. Surgical trauma triggers a stress response that raises the patient's renin-angiotensin levels and fluctuates his or her blood pressure considerably. Intraoperative traction will also increase sympathetic nerves tension and aggravate coronary spasm, so patients with esophageal and lung cancer are more likely to have arrhythmia after surgery [23], which is not conducive to their perioperative recovery. In order to improve the symptoms of arrhythmia patients, sodium channel blockers, calcium channel blockers, and other drugs are often used clinically.

In Chinese medicine, the clinical symptoms of patients with arrhythmia are classified as “chest paralysis” and “palpitation.” The main cause of the disease is weakness, lack of innate endowment, or excessive thinking, or invasion of external evil, depletion of heart qi, deficiency of heart qi, the heart's main blood vessels and the function of hiding the spirit, blocking the qi, inducing chest tightness and shortness of breath, and spontaneous sweating. The disease is induced by the deficiency of Qi and blood over time, and the deficiency of blood does not nourish the heart. Yangxin Yiqi Tongmai decoction is based on the addition and subtraction of the clinical symptoms of patients on the basis of pulse-activating decoction and grilled Glycyrrhiza decoction and Cassia Twig and Dragon Bone Combination. The monarch medicines in the prescription are *Panax quinquefolium* and *Salvia miltiorrhiza*. *Panax quinquefolium* tonifies Qi and nourishes Blood, while *Salvia miltiorrhiza* invigorates blood to regulate menstruation, dispel blood stasis, and relieve pain. The combination of the two drugs is effective in tonifying Qi and nourishing blood, invigorating blood, and dispelling blood stasis. Semen Ziziphi Spinosae, Radix Puerariae, Taxillus chinensis Danser, Rhizoma Nardostachyos, and Coptidis Rhizoma are used together to calm the mind and tranquilize the spirit, raise and lower the qi in a measured manner, and nourish the essence and blood [24]. Many clinical studies have demonstrated that herbal medicines combined with western medicines can better relieve the symptoms of patients with cardiac arrhythmias.

Cedilan is a commonly used digitalis drug in clinical practice, which can reduce the heart rate and strengthen the myocardial contractile function of patients, which is of high value in paroxysmal supraventricular tachycardia. However, cedilan, similar to other digitalis drugs, can easily cause gastrointestinal reactions. Some patients also suffer from neurological complaints, such as dizziness, insomnia, and depression. In severe cases, digitalis toxicity may even aggravate cardiac arrhythmias. Therefore, it should be used with caution. In a study by Fonseca L scholars et al., the onset of action of sildiran for arrhythmias in heart failure was significantly longer than that of amiodarone treatment [25]. This study also investigated and concluded the same result, indicating that amiodarone has a faster effect then the cedilan, and the patient's average ventricular rate decreased more significantly [26, 27].

At present, the latest version of the arrhythmia treatment guidelines has recommended amiodarone as the first-line treatment for electric shock to reverse arrhythmia [28]. The drug is a beta-adrenergic receptor blocker, which can prolong the action potential of myocardial tissue and reduce re-entrant excitation. It can avoid rapid sodium influx in atrial and myocardial conduction, which can effectively control hemodynamic changes and reduce blood pressure fluctuations in patients. Therefore, the stress indicators and blood pressure levels of the observation group after the treatment are remarkably better than those of the control group. Taken together, amiodarone can inhibit factors that predispose to arrhythmias. In addition, amiodarone exhibited no inhibitory effect on left ventricular function and can be used to alleviate arrhythmic patients with severe left ventricular insufficiency [29]. For some patients with preoperative circulatory and respiratory dysfunction, amiodarone can also improve its cardiopulmonary function. It has been found that the heart function indexes of the observation group after treatment were considerably better than those of the control group, indicating that the effect of amiodarone was superior to that of the cedilan [30]. The analysis of the results revealed that amiodarone is a class III antiarrhythmic drug with the presence of mild noncompetitive alpha and beta-adrenergic receptor blockers. Its ability to prolong the action potential and effective inactivity of myocardial tissues at various sites can eliminate fold excitation. It reduces conduction velocity by inhibiting Na+ inward flow in atrial and myocardial conduction fibers. It does not adversely affect the resting membrane potential and action potential height and inhibits the antegrade conduction of the atrioventricular bypass more than the retrograde. Prolongation of the Q-T interval and T-wave changes may occur on the ECG due to excessive prolongation of repolarization. With amiodarone, its ability to effectively inhibit adrenergic receptors allows for a decrease in sympathetic activity, which in turn improves arrhythmic conditions [31, 32].

Chen et al. showed that amiodarone exerted little effect on arrhythmias, intraventricular conduction, either by increasing the pacing threshold. In addition, the drug is metabolized mainly by the hepatic cytochrome P450 system with little renal clearance, and thus it does not increase the renal burden of patients [33]. A large number of studies have confirmed that amiodarone bears a higher safety and a lower probability of adverse reactions [34]. This study found that the adverse reactions of the two groups of patients were mostly dizziness and fatigue and gastrointestinal reactions. The observation group had significantly lower adverse reactions rate than the control group, suggesting that it can be used in middle-aged and elderly patients with lung and esophageal cancer whose body function and immune abilities are gradually declining, and it is beneficial to reduce the body burden of patients [35]. The reason may be that amiodarone is a class III antiarrhythmic drug with both mild class I and class IV antiarrhythmic properties and is a broad-spectrum antiarrhythmic drug. After oral administration, 62.1% binds to albumin in plasma, and 33.5% may bind to *β*-lipoprotein, so its oral effect is slow. The bioavailability of amiodarone is on average around 50%. Not only can amiodarone treat arrhythmias in the elderly but long-term use of amiodarone in small doses can also serve the purpose of controlling arrhythmias and consolidating the therapeutic effect. The patients had arrhythmic manifestations effectively controlled, and myocardial oxygen consumption was significantly reduced, and therefore, myocardial cell function was significantly restored, and cardiac function was obviously enhanced [36, 37].

This trial is instructive, but the following problems remain: small sample size, short observation period, and no long-term follow-up. Despite some drawbacks, the method can be applied to treat patients with cerebral aneurysms in various medical institutions. It is expected that in the future, a large number of investigators and patients will cooperate and conduct clinical studies together with larger samples to provide more clinical evidence for the study and application of this method.

## 5. Conclusions

In this study, we explored the effect of amiodarone and cedilan in the treatment of patients with arrhythmia after esophageal and lung cancer. It has been observed that amiodarone can alleviate the stress state of patients with arrhythmia after esophageal and lung cancer surgery, stabilize the blood pressure indicators, and improve arrhythmia symptoms. Our findings are worthy of promotion and application in clinical practice.

## Figures and Tables

**Figure 1:** Intergroup comparison of treatment effects (*n*(%)). Note: see Figures 1(a) and 1(b) for the observation group and the control group, respectively. The black area in the figure refers to markedly effective, the dark gray area means effective, and the light gray area indicates ineffective. # means *P* < 0.05. In the observation group, 15 (50.0%), 13 (43.3%), and 2 (6.7%) patients were markedly effective, effective, and ineffective after the treatment, and in the control group, 8 (26.7%), 12 (40.0%), and 10 (33.3%) patients were remarkably effective, effective, and ineffective after treatment, respectively.

**Figure 2:** Intergroup comparison of average ventricular rate before and after treatment ($\bar{x}$ ± *s*, times/min). Note: the horizontal axis in Figure 2 is from left to right before and after treatment, and the vertical axis is the average ventricular rate (times/min). The dotted line in the figure refers to the observation group and the square line the control group. # indicates *P* < 0.001. There was no significant difference in the average ventricular rate before treatment between the observation group and the control group (148.65 ± 12.65 vs 148.54 ± 12.45 and *P* > 0.05). The average ventricular rate after treatment was notably lower in the observation group than the control group (80.65 ± 8.65 vs 101.54 ± 10.11 and *P* < 0.001).

**Figure 3:** Intergroup comparison of drug onset time ($\bar{x}$ ± *s* min). Note: in Figure 3, the horizontal axis is the observation group and the control group from left to right, and the vertical axis is the drug onset time (min). # indicates *P* < 0.001. The drug onset time was obviously lower in the observation group as compared to the control group (18.54 ± 2.15 vs 32.14 ± 3.98 and *P* < 0.001).

**Figure 4:** Intergroup comparison of stress indicators ($\bar{x}$ ± *s*). Note: the horizontal axes of Figures 4(a) and 4(b) are pretreatment and post-treatment, respectively, from left to right. The black area in the figure means the observation group, and the gray area indicates the control group. # indicates *P* < 0.001. See Figure (a) for the blood glucose level. The blood glucose level was significantly lower in the observation group after treatment than the control group (3.89 ± 0.32 vs 5.42 ± 0.68, *P* < 0.001). Figure (b) indicates the insulin level. After treatment, the insulin level was significantly higher in the observation group than the control group (14.20 ± 1.65 vs 11.10 ± 1.20, *P* < 0.001).

**Table 1:** Intergroup comparison of general data.

Group	Observation group (*n* = 30)	Control group (*n* = 30)	*X* ^2^/*t*	*P*
Gender			0.617	0.432
Male	16	19		
Female	14	11		

Age (year old)				
Age range	43–77	42–77		
Mean age	63.50 ± 6.88	63.60 ± 9.66	0.046	0.963

Mean weight (kg)	56.21 ± 2.15	56.23 ± 2.66	0.032	0.975
BMI (kg/m^2^)	23.45 ± 3.15	23.50 ± 3.20	0.061	0.952

Type of disease			0.272	0.602
Esophageal cancer	12	14		
Lung cancer	18	16		

Marital status			0.111	0.739
Married	25	24		
Single	5	6		

Medical expenses payment method				
Medical insurance	15	14	0.067	0.796
Commercial insurance	10	10	0.000	1.000
Others	5	6	0.111	0.739

Place of residence			0.067	0.795
Township	14	13		
Countryside	16	17		

Monthly income (yuan)			0.067	0.796
≥4000	15	14		
<4000	15	16		

Living habits				
History of smoking	12	13	0.069	0.793
Drinking history	14	12	0.272	0.602

Education level			0.069	0.793
High school and below	18	17		
University and above	12	13		

**Table 2:** Intergroup comparison of cardiac function indexes ($\bar{x}$ ± *s*).

	Observation group		Control group		*t*	*P*
LVEDD (mm)	Pretreatment	65.47 ± 5.98	Pretreatment	65.40 ± 5.48	0.047	0.963
	Post-treatment	50.12 ± 5.10	Post-treatment	56.98 ± 5.45	5.034	<0.001
	*T*	10.697	*t*	5.967		
	*P*	<0.001	*P*	<0.001		

LVEF (%)	Pretreatment	45.68 ± 6.98	Pretreatment	45.47 ± 6.51	0.121	0.905
	Post-treatment	62.45 ± 5.98	Post-treatment	55.65 ± 5.68	4.516	<0.001
	*t*	9.993	*t*	6.454		
	*P*	<0.001	*P*	<0.001		

SV (L/min)	Pretreatment	3.25 ± 0.65	Pretreatment	3.28 ± 0.57	0.190	0.850
	Post-treatment	4.98 ± 0.87	Post-treatment	4.25 ± 0.88	3.231	0.002
	*T*	8.725	*t*	5.067		
	*P*	<0.001	*P*	<0.001		

**Table 3:** Intergroup comparison of the incidence of adverse reactions (*n* (%)).

Group	Dizziness and fatigue	Gastrointestinal reaction	Increased creatinine	Increased blood phosphorus	Total incidence
Observation group	1 (3.3)	1 (3.3)	0 (0.0)	0 (0.0)	2 (6.7)
Control group	2 (6.7)	4 (13.3)	2 (6.7)	2 (6.7)	10 (33.3)
*X* ^2^	0.351	1.964	2.069	2.069	6.667
*P*	0.554	0.161	0.150	0.150	0.010

**Table 4:** Intergroup comparison of blood pressure levels ($\bar{x}$ ± *s* and mmHg).

	Observation group		Control group		*t*	*P*
Systolic blood pressure	Pretreatment	156.65 ± 15.32	Pretreatment	156.78 ± 15.24	0.033	0.974
	Post-treatment	143.98 ± 12.68	Post-treatment	150.74 ± 12.68	2.065	0.043
	*t*	3.490	*t*	1.669		
	*P*	0.001	*P*	0.101		

Diastolic blood pressure	Pretreatment	90.26 ± 8.12	Pretreatment	90.20 ± 8.10	0.029	0.977
	Post-treatment	80.45 ± 5.98	Post-treatment	88.65 ± 7.98	4.504	<0.001
	*t*	5.328	*t*	0.747		
	*P*	<0.001	*P*	0.458		

## Data Availability

The data used to support the findings of this study are available from the corresponding author upon request.
